# Therapeutic Effect of Laparoscopic Cholecystectomy on Patients with Cholecystolithiasis Complicated with Chronic Cholecystitis and Postoperative Quality of Life

This article has been retracted.

**DOI:** 10.1155/2022/6813756

**Published:** 2022-07-21

**Authors:** Jie Song, Jie Chen, Chunyan Lin

**Affiliations:** ^1^Department of General Surgery, Affiliated Hospital of Jiangnan University, Wuxi, China; ^2^Department of Hepatobiliary Surgery, Affiliated Hospital of Jiangnan University, Wuxi, China

## Abstract

**Objective:**

To assess the treatment outcome and postoperative quality of life of patients with gallbladder stones and chronic cholecystitis after open cholecystectomy and laparoscopic cholecystectomy.

**Methods:**

Between 2018 and 2020, 108 patients with gallbladder stones and chronic cholecystitis treated in our hospital were assessed for eligibility and randomly recruited. They were concurrently assigned (1 : 1) to receive either open cholecystectomy (control group) or laparoscopic cholecystectomy (study group). Outcome measures include surgical indices, inflammatory response, postoperative complications, and quality of life of patients.

**Results:**

Laparoscopic cholecystectomy was associated with a shorter duration of surgery, intraoperative bleeding, time to first postoperative bowel movement, and postoperative hospital stay versus open cholecystectomy (*P* < 0.05). The levels of inflammatory factors of all eligible patients were comparable before cholecystectomy (*P* > 0.05). The patients given laparoscopic cholecystectomy showed lower levels of C-reactive protein (CRP), interleukin (IL)-6, and IL-8 versus those given open cholecystectomy (*P* < 0.05). Laparoscopic cholecystectomy resulted in a significantly lower incidence of complication (3.56%) versus open cholecystectomy (24.07%) (*P* < 0.05). The patients had significantly higher physical, psychological, and social function scores after laparoscopic cholecystectomy versus open cholecystectomy (*P* < 0.05).

**Conclusion:**

Laparoscopic cholecystectomy provides better surgical results, mitigates the inflammatory response, lowers the incidence of complications, and improves the quality of life of patients versus open cholecystectomy, so it is worthy of application in clinical treatment.

## 1. Introduction

Chronic cholecystitis is a chronic inflammatory lesion of the digestive system, which is a chronic inflammation of the gallbladder elicited by various causes such as recurrent acute or subacute cholecystitis or long-standing gallstones [1]. The prevalence of chronic cholecystitis in adults is reported to be 0.78% to 3.91% in China, and the prevalence of gallbladder stones is 2.3% to 6.5% [2]. The prevalence of gallbladder stones is higher in women than in men, and the peak incidence is after the age of 50. As the standard of living of the Chinese people continues to improve, the incidence of chronic cholecystitis is on the rise [3]. Its early clinical symptoms mainly include abdominal pain, belching, vomiting, and other symptoms of hepatogenic dyspepsia [4]. Complications occur most often in acute attacks of cholecystitis and pancreatitis, and about 25% of patients develop bacterial infections, caused by obstruction of the cystic duct or common bile duct, which seriously endanger the health and daily life of the patient. Most patients with chronic cholecystitis are accompanied by gallbladder stones, also known as cholelithiasis [5], a condition in which stones are found in the biliary system, such as the gallbladder or bile ducts, with the typical symptoms of biliary colic. Epidemiological data show that nearly 70% of patients with chronic cholecystitis have gallbladder stones; therefore, the combination of chronic cholecystitis with gallbladder stones has received much attention in recent years, and timely and effective interventions are essential to improve the outcome and prognosis of patients' lives [6–8].

Oral lithotripsy may be considered in symptomatic patients who are not candidates for surgery and have cholesterol stones assessed by abdominal ultrasonography as having normal gallbladder function and negative radiographs [9]. Ursodeoxycholic acid (UDCA) is currently the only bile acid drug approved by the US FDA for the nonsurgical treatment of gallstones [10]. Patients with chronic cholecystitis often suffer from dyspepsia, and in the early stages of dyspepsia, medications such as azintamide or other pancreatic enzymes can be used to improve the symptoms [11]. Patients with chronic cholecystitis usually do not require antibiotics. However, it is important to use antibiotics appropriately when the patient has a combination of underlying diseases, especially if there is impairment of liver or kidney function [12]. However, when surgery is indicated, surgical removal of the gallbladder is the treatment of choice [13]. Cholecystectomy is the most common procedure in biliary surgery for various acute and chronic cholecystitis, symptomatic gallbladder stones, and gallbladder augmentation lesions, and its long-term outcomes are considered satisfactory in most cases. Cholecystectomy consists of open cholecystectomy and laparoscopic cholecystectomy [14–16]. With advances in medical technology, both surgical procedures are effective in the treatment of patients with gallbladder stones combined with chronic cholecystitis, but comparative analyses of their treatment outcomes and postoperative quality of life are inadequate due to the lack of standardized and universally validated tools [17].

Accordingly, the present study was to assess the treatment outcome and postoperative quality of life of patients with gallbladder stones and chronic cholecystitis after open cholecystectomy and laparoscopic cholecystectomy to provide a reference for clinical surgical alternatives.

## 2. Materials and Methods

### 2.1. Research Subjects

Between 2018 and 2020, 108 patients with gallbladder stones and chronic cholecystitis treated in our hospital were assessed for eligibility and randomly recruited. They were concurrently assigned (1 : 1) to a control group or a study group. The study/research was approved by the Ethics Committee of the Affiliated Hospital of Jiangnan University, No. j29879.

### 2.2. Inclusion and Exclusion Criteria

#### 2.2.1. Inclusion Criteria

1. All diagnosed with gallbladder stones and chronic cholecystitis [18]
2. With consciousness and no combined psychiatric diseases
3. With no autoimmune system diseases or acute biliary pancreatic diseases

#### 2.2.2. Exclusion Criteria

1. With cardiac, hepatic, renal, and other important organ insufficiencies
2. With surgical-related contraindications
3. With coagulation disorders

### 2.3. Methods

Patients in both groups were in the supine position. Open cholecystectomy was performed for patients in the control group [19]. After general anaesthesia, a 10 cm long incision is made in the right upper abdomen through the rectus abdominis muscle. The abdominal wall is incised into the abdominal cavity in sequence, and the operation is extended with a large “S” shaped hook. The gallbladder is removed in a cisreverse fashion, the exudate is aspirated with sterile gauze, a drainage tube is placed in the abdominal wall, the abdominal cavity is cleaned, and the incision is closed layer by layer. Postoperative gastrointestinal decompression and antiinfective treatments were given. The patients in the study group underwent laparoscopic cholecystectomy [7]. The patient was given intravenous general anaesthesia with tracheal intubation preoperatively, and a 1 cm curved incision was made below the umbilicus after the routine establishment of a CO_2_ pneumoperitoneum, followed by the placement of a 10 mm Trocar to examine the abdominal cavity condition. A 1 cm incision was made 4 cm below the glabella as the main operating port, where a 10 mm Trocar was placed. A 5 mm Trocar was placed 2 cm below the right rib in the anterior axillary line and 2 cm below the rib in the right midclavicular line to establish a secondary operating port, and the gallbladder and the cystic duct were fully exposed and separated. The gallbladder was resected under laparoscopic assistance and removed through the main operating port. The surgical area was irrigated, and the incision was sutured sequentially. Postoperatively, routine gastrointestinal decompression and anti-infective treatment were given.

### 2.4. Outcome Measures

① Surgical indices: the surgical conditions (including the duration of surgery, intraoperative bleeding, time to first postoperative bowel movement, and postoperative hospital stay) of the two groups were recorded and compared.
② Inflammatory factors: fasting venous blood was collected before and 2 d after surgery in the two groups, respectively, to separate serum. Serum C-reactive protein (CRP) was determined by the scattering turbidimetric method, and interleukin-6 (IL-6), and interleukin-8 (IL-8) were determined by the enzyme-linked immunosorbent assay (EusA).
③ Complications: the occurrence of surgical complications (including incisional infection, bile duct bleeding, abdominal infection, pulmonary infection, and intrahepatic cholestasis) was recorded separately in both groups to calculate the incidence. Complication rate = number of people with complications/total number of people × 100%.
④ Quality of life [20]: the quality of life of the two groups was analysed by comparing the scores of the 3 domains of physical function, psychological function, and social function of the patients. Each dimension had 5 assessment factors, and the scores were proportional to the quality of life.

### 2.5. Statistical Analysis

SPSS 22.0 software was used for data analyses. The count data were expressed as (*n* (%)) and processed using the chi-square test, and the measurement data were expressed as ($\bar{x}$ ± *s*) and processed using the *t*-test. Differences were considered statistically significant at *P* < 0.05.

## 3. Results

### 3.1. Baseline Information

The baseline characteristics of the patients in the study group (28 males and 26 females, aged 58–77 years, mean age of (59.23 ± 3.78) years, duration of disease of [1–5] years, mean duration of disease of (3.02 ± 0.82) years, the stone diameter of (2.87–18.67) mm, and mean diameter of (5.23 ± 2.17) mm) were comparable with those in the control group (27 males and 27 females, aged 55–79 years, mean age of (59.18 ± 4.05) years, duration of disease of [1–5] years, mean duration of disease of (3.18 ± 0.65) years, the stone diameter of (3.25–20.02) mm, and mean diameter of 5.48 ± 1.99 mm) (*P* > 0.05) (Table 1).

### 3.2. Surgical Conditions

Compared to open cholecystectomy (120.98 ± 31.65, 119.16), laparoscopic cholecystectomy was associated with shorter operative time, intraoperative bleeding, time to first postoperative bowel movement, and postoperative hospital stay (88.25 ± 25.63, 75.83 ± 7.23, 37.85 ± 3.17, 5.02 ± 3.21) ± 14.41, 58.25 ± 5.21, 8.74 ± 3.11) (*P* < 0.05) (Table 2).

### 3.3. Inflammatory Response

All eligible patients had comparable levels of inflammatory factors prior to cholecystectomy (*P* > 0.05). CRP, IL-6, and IL-8 levels were lower in laparoscopic cholecystectomy patients (16.18 ± 3.21, 55.74 ± 6.18, 22.57 ± 5.67) than in open cholecystectomy patients (26.24 ± 2.87, 64.87 ± 4.96, 41.68 ± 5.21) (*P* < 0.05) (Table 3).

### 3.4. Complications

Compared with open cholecystectomy, laparoscopic cholecystectomy had a significantly lower complication rate (3.56%) (1 (1.85%) incisional infection, 1 (1.85%) bile duct haemorrhage, and 1 (1.85%) intrahepatic cholestasis) and (24.07%) (5 (9.25%) incisional infections, 2 (3.71%) bile duct haemorrhages, 1 (1.85%) abdominal infection) cases, 1 (1.85%) pulmonary infection, 4 (7.41%) cases of intrahepatic cholestasis) (*P* < 0.05) (Table 4).

### 3.5. Quality of Life

Patients' physical, psychological, and social functioning scores were significantly higher after laparoscopic cholecystectomy (86.23 ± 5.96, 87.45 ± 5.12, and 83.17 ± 4.91) than after open cholecystectomy (73.84 ± 5.17, 76.77 ± 4.84, and 73.65 ± 5.95) (*P* < 0.05) (Table 5).

## 4. Discussion

Patients with gallbladder disease usually present with a long duration, acute and rapid progression, and are highly susceptible to various complications if not treated promptly. Long-term episodes of acute or subacute cholecystitis may lead to chronic cholecystitis disease. Gallbladder stones are the main cause of chronic cholecystitis. Stones can lead to repeated obstruction of the gallbladder duct, causing damage to the gallbladder mucosa, resulting in recurrent inflammatory responses in the gallbladder wall, scar formation, and gallbladder dysfunction [21]. Chronic nonlithiatic cholecystitis is mainly caused by bacterial infections of enteric origin, where intestinal bacteria can pass through the bile duct to the gallbladder, or through the blood or lymphatic route to the gallbladder [22]. The treatment of patients with cholecystitis combined with gallstones was mostly performed by open surgery previously [23], which could achieve satisfactory therapeutic results but is associated with disadvantages such as significant trauma, long operative time, large intraoperative blood volume, and a negative impact on patients' gastrointestinal function [24]. In recent years, laparoscopic cholecystectomy has been widely used in the clinical treatment of patients with chronic cholecystitis and gallbladder stones [25, 26]. As the gold standard for the treatment of gallbladder disease, laparoscopic cholecystectomy has the advantages of being minimally invasive, small incision, less pain, and quicker postoperative recovery, and is conducive to preserving the contractile function of the gallbladder [27, 28]. In recent years, extensive research has been undertaken on the treatment of gallbladder stones and chronic cholecystitis [29].

The results of this study showed that laparoscopic cholecystectomy was associated with shorter operative time, intraoperative bleeding, time to first postoperative bowel movement, and shorter postoperative hospital stay compared to open cholecystectomy (*P* < 0.05), suggesting the advantages of laparoscopic cholecystectomy. This was attributed to the clear laparoscopic view of the gallbladder surface and surrounding tissues. The clear surgical view combined with the advanced endoscopic equipment maximises the noninvasive nature of the human tissue and speeds up postoperative recovery. The patients given laparoscopic cholecystectomy showed lower levels of CRP, IL-6, and IL-8 versus those given open cholecystectomy (*P* < 0.05), indicating that laparoscopic cholecystectomy results in less trauma and a milder inflammatory response. The reason for this is that open cholecystectomy is highly invasive and has a greater impact on the patient's tissues, endocrine system, and associated cytokines, whereas laparoscopic cholecystectomy has a small surgical incision, a low incidence of bile duct injury, and a low incidence of bile leakage from the stump. The gallbladder duct is delayed, and there is less postoperative intraabdominal bleeding and less interference with organ function. In addition, laparoscopic cholecystectomy had a significantly lower complication rate and a significantly higher quality of life score compared to open cholecystectomy (*P* < 0.05). The cure rate of laparoscopic cholecystectomy exceeded 98%, with no absolute contraindications, small surgical incisions, and rapid postoperative recovery, reducing the incidence of postoperative complications and improving the quality of life of patients. Investigated the clinical efficacy of laparoscopic cholecystectomy versus open cholecystectomy and found that laparoscopic cholecystectomy is characterized by less trauma, less body impact, and faster post-operative recovery versus open cholecystectomy, which is consistent with the results of the present study.

Chronic cholecystitis belongs to the category of hypochondriac pain in TCM, with the disease located in the gallbladder and liver in a close relationship, often accompanied by liver qi stagnation, liver and gallbladder dampness and heat, stasis, and blood blockage [30]. Drugs such as Chai Hu to clear the liver, Yu Jin to clear heat and dampness, Chuan Xiong to activate blood circulation and remove blood stasis, Qian Cao and Cang Zhu to clear heat and dampness, Bai Shao to soften the liver and relieve pain, Yuan Hu Suo to move Qi and blood to relieve pain, Hai Jin Sha to clear heat and dampness and drain stones, and Citrus Aurantium to broaden the middle and move Qi to facilitate the draining of liver Qi [31]. Different prescriptions should be used according to the type of Chinese medicine, and it should be emphasized that in the actual symptoms of chronic cholecystitis, the main focus is on eliminating evil, such as clearing heat and dampness, soothing the liver and bile, and moving Qi and invigorating blood, while in the deficiency symptoms, the main focus is on helping the righteous, such as strengthening the spleen and benefiting Qi, nourishing Yin and softening the liver, and can also be combined with Chinese medicine specialties, such as acupuncture and moxibustion ear points, medication paste on the abdomen, and acupoint burial [30–32].

But our experiments still have limitations. First of all, we need long-term regular follow-up visits to determine the prognostic effect. Second, we need to expand the scope of the trial and the sample size. Although sensitive and responsive instruments exist for measuring the quality of life after cholecystectomy, more research is needed to identify modifications that may lead to significant improvements.

## 5. Conclusion

To sum up, laparoscopic cholecystectomy provides better surgical results, mitigates the inflammatory response, lowers the incidence of complications, and improves the quality of life of patients versus open cholecystectomy, so it is worthy of application in clinical treatment.

## Figures and Tables

**Table 1:** Comparison of baseline characteristics ($\bar{x}$ ± *s*).

Groups	*n*	Gender (male/female)	Age (year)	Mean age (year)	Duration of disease (year)	Mean duration of disease (year)	Stone diameter (cm)	Mean diameter (cm)
Study group	54	28/26	58–77	59.23 ± 3.78	1–5	3.02 ± 0.82	2.87–18.67	5.23 ± 2.17
Control group	54	27/27	55–79	59.18 ± 4.05	1–5	3.18 ± 0.65	3.25–20.02	5.48 ± 1.99
*t* value	—	—	—	0.066	—	1.124	—	0.624
*P* value	—	—	—	0.948	—	0.264	—	0.534

**Table 2:** Comparison of surgical conditions ($\bar{x}$ ± *s*).

Groups	*n*	Duration of surgery (min)	Intraoperativebleeding volume (ml)	Time to first post-operativebowel movement (h)	Postoperativehospital stay (d)
Study group	54	88.25 ± 25.63	75.83 ± 7.23	37.85 ± 3.17	5.02 ± 3.21
Control group	54	120.98 ± 31.65	119.16 ± 14.41	58.25 ± 5.21	8.74 ± 3.11
*t* value	—	5.906	19.750	24.581	6.116
*P* value	—	＜0.001	＜0.001	＜0.001	＜0.001

**Table 3:** Comparison of inflammatory factors levels ($\bar{x}$ ± *s*).

Groups	*n*	CRP (mg/L)		IL-6 (mg/L)		IL-8 (mg/L)	
		Before treatment	After treatment	Before treatment	After treatment	Before treatment	After treatment
Study group	54	6.25 ± 1.98	16.18 ± 3.21	46.21 ± 5.34	55.74 ± 6.18	10.17 ± 3.74	22.57 ± 5.67
Control group	54	6.11 ± 2.06	26.24 ± 2.87	46.18 ± 5.29	64.87 ± 4.96	10.23 ± 3.65	41.68 ± 5.21
*t* value	—	0.360	17.168	0.029	8.467	0.084	18.237
*P* value	—	0.720	＜0.001	0.977	＜0.001	0.933	＜0.001

**Table 4:** Comparison of complications (%).

Groups	*n*	Incisional infection	Bile duct bleeding	Abdominal infection	Pulmonary infection	Intrahepatic cholestasis	Incidence
Study group	54	1 (1.85)	1 (1.85)	0 (0.00)	0 (0.00)	1 (1.85)	3 (5.56)
Control group	54	5 (9.25)	2 (3.71)	1 (1.85)	1 (1.85)	4 (7.41)	13 (24.07)
*x* ^2^ value	—	—	—	—	—	—	7.337
*P* value	—	—	—	—	—	—	0.007

**Table 5:** Comparison of quality of life ($\bar{x}$ ± *s*).

Groups	*n*	Physical function	Psychological function	Social function
Study group	54	86.23 ± 5.96	87.45 ± 5.12	83.17 ± 4.91
Control group	54	73.84 ± 5.17	76.77 ± 4.84	73.65 ± 5.95
*t* value	—	11.540	11.139	9.069
*P* value	—	＜0.001	＜0.001	＜0.001

## Data Availability

All data generated or analysed during this study are included in this published article.
